The article "Epigenetic silenced miR‐125a‐5p could be self‐activated through targeting Suv39H1 in gastric cancer" was retracted in 2021. Reasons: errors in the data; errors in the images; unreliable results or conclusions; concerns about a third party's involvement.

# Epigenetic silenced miR‐125a‐5p could be self‐activated through targeting Suv39H1 in gastric cancer

**DOI:** 10.1111/jcmm.13716

**Published:** 2018-08-17

**Authors:** Mingzhi Cai, Qiuxian Chen, Juntao Shen, Chenbing Lv, Lisheng Cai

**Affiliations:** ^1^ Department of General Surgery Zhangzhou Affiliated Hospital of Fujian Medical University Zhangzhou City China

**Keywords:** epigenetic silence, gastric cancer, miR‐125a‐5p, Suv39H1

## Abstract

Emerging evidence suggests that microRNAs (miRNAs) serve an important role in tumorigenesis and development. Although the low expression of miR‐125a‐5p in gastric cancer has been reported, the underlying mechanism remains unknown. In the current study, the low expression of miR‐125a‐5p in gastric cancer was verified in paired cancer tissues and adjacent non‐tumour tissues. Furthermore, the GC islands in the miR‐125a‐5p region were hypermethylated in the tumour tissues. And the hypermethylation was negatively correlated with the miR‐125a‐5p expression. Target gene screening showed that the histone methyltransferase Suv39H1 was one of the potential target genes. In vitro studies showed that miR‐125a‐5p could directly suppress the Suv39H1 expression and decrease the H3K9me3 levels. On the other hand, the Suv39H1 could induce demethylation of miR‐125a‐5p, resulting in re‐activation of miR‐125a‐5p. What is more, overexpessing miR‐125a‐5p could also self‐activate the silenced miR‐125a‐5p in gastric cancer cells, which suppressed cell migration, invasion and proliferation in vitro and inhibited cancer progression in vivo. Thus, we uncovered here that the epigenetic silenced miR‐125a‐5p could be self‐activated through targeting Suv39H1 in gastric cancer, suggesting that miR‐125a‐5p might be not only the potential prognostic value as a tumour biomarker but also potential therapeutic targets in gastric cancer.

## 1 INTRODUCTION

Gastric cancer is still the fourth most common cancer all over the world and the second most universal cause of cancer death globally, although there has been a constant descent in morbidity and mortality in the past few decades.^1^ The early clinical inspection of gastric cancer was under 15%, and cases of advanced gastric cancer accounted for 85%.^2^ At present, the primary treatment choices are surgical intervention, chemotherapy, immunogene therapy and target therapy. The clinical result of gastric cancer mainly depends on the stage of tumour. Unfortunately, gastric cancer patients’ median survival time is no more than 6‐9 months.^3^ It is unlimited proliferation of cancer cells and ability of intense invasive and metastasis that mainly causes high malignancy degree and poorer survival time. As a result, a novel diagnostic means and improved prognosis of gastric cancer might be created through identification of molecular aberrations, which can predict cancer progression and survival rate.

The article "Epigenetic silenced miR‐125a‐5p could be self‐activated through targeting Suv39H1 in gastric cancer" was retracted in 2021. Reasons: errors in the data; errors in the images; unreliable results or conclusions; concerns about a third party's involvement.

An increasing number of evidence shows that various miRNAs, a novel class of small (20‐24 nucleotides) non‐coding regulatory RNAs, are related with tumour formation, development, progression and the responses to the treatment,^4^, ^5^, ^6^ including the gastric cancer.^3^, ^7^, ^8^ Among all the dysregulated miRNAs, miR‐125a‐5p is one of the most down‐regulated or mutated miRNAs in gastric cancer tissues.^9^

A number of studies have shown that the microRNA‐125a‐5p is an important tumour suppressor, and its expression is reduced in many types of human cancer, including in laryngeal cancer,^10^ juvenile angiofibromas,^11^ colorectal cancer,^12^ breast cancer,^13^, ^14^ lung cancer,^15^, ^16^, ^17^ cervical carcinomas,^18^ prostate and pancreatic cancers.^19^ MicroRNA‐125a‐5p has been demonstrated as an independent prognostic factor in gastric cancer and inhibiting the gastric cancer development,^20^ through targeting oncogenes such as vascular endothelial growth factor A^21^ and E2F transcription factor 3.^22^ Overexpressing miR‐125a‐5p could inhibit the cancer proliferation and migration.^23^, ^24^

However, the underlying mechanism of the low expression of miR‐125a‐5p in gastric cancer remains unknown. It has been demonstrated that some epigenetic modulators could modulate the miR‐125‐5p expression, such as HDACs (histone deacetylases),^13^, ^25^ or be modulated by miR‐125‐5p, such as Sirtuins.^26^ Furthermore, the putative promoter regions the miR‐125a‐5p are embedded in CpG islands and are hypermethylated in glioma cells.^27^ Considering the above findings, we wanted to test the expression and methylation status of miR‐125a‐5p in gastric cancer tissues and adjacent non‐tumour tissues and then to evaluate whether DNA methylation participates in regulating miR‐125a‐5p expression in human gastric cancer.

In this study, it was confirmed that the miR‐125a‐5p expression was reduced in most gastric cancer tissues comparing with the adjacent non‐tumour tissues. DNA methylation analysis showed the miR‐125a‐5p promoter was highly methylated and negatively associated its expression. Target gene screening and validation showed that the histone methyltransferase Suv39H1 was the miR‐125a‐5p target gene, which was also involved into the epigenetic silencing of the miR‐125a‐5p. Overexpessing miR‐125a‐5p could self‐activate the silenced miR‐125a‐5p in gastric cancer cells, resulting in cancer suppression in vitro and in vivo. The data here showed that the miR‐125a‐5p might be not only the potential prognostic value as a tumour biomarker but also potential therapeutic targets in gastric cancer.

The article "Epigenetic silenced miR‐125a‐5p could be self‐activated through targeting Suv39H1 in gastric cancer" was retracted in 2021. Reasons: errors in the data; errors in the images; unreliable results or conclusions; concerns about a third party's involvement.

## 2 METHODS AND MATERIALS

### 2.1 Patients

The clinical characteristics of all 286 patients in our study are listed in Table 1. Gastric tissues were obtained from gastric cancer patients undergoing gastric resection at the Zhangzhou Affiliated Hospital of Fujian Medical University. Patients with a previous history of another primary tumour, or those who had previously received chemotherapy and/or radiotherapy were excluded from the study. Written consent was obtained prior to surgery. The study was approved by the Ethics Committee of Zhangzhou Affiliated Hospital of Fujian Medical University. The cancer tissues and adjacent non‐tumour tissues were quickly separated into two sections following resection. One was immediately frozen in liquid nitrogen for RNA and DNA isolation and another was fixed in formalin for pathological examination. Final pathological diagnosis was independently made by at least two professional pathologists.

**Table 1:** Clinicopathological features and miR‐125a‐5p expression

	N	miR‐125a‐5p expression in tumour		*P* value
		Low (n = 210)	High (n = 76)	
Age, y				
<65	214	159	55	.913
≥65	72	51	21	
Gender				
Male	110	78	32	.382
Female	176	132	44	
Tumour size, cm				
<50 mm (small)	124	64	60	.001^a^
≥51 mm (large)	162	146	16	
Differentiation				
Well	31	14	17	.126
Moderate	122	74	48	
Low	133	85	48	
Lymph node metastasis				
Yes	138	132	6	.009^a^
No	148	78	70	
Liver metastasis				
Yes	128	123	5	.012^a^
No	158	87	71	

a *P *<* *.05 indicates a significant association among the variables.

### 2.2 RNA isolation and RT‐qPCR

Total RNA from tissues or cultured cells was isolated using TRIzol reagent (Thermo Fisher Scientific) according to the manufacturer's protocol. RNA concentration was measured using NanoDrop ND‐1000 (Thermo Fisher Scientific), and the quality was assessed using electrophoresis with 1.5% denaturing agarose gels. TaqMan probe‐based qPCR was performed using a commercial kit (Applied Biosystems, Thermo Fisher Scientific) according to the manufacturer's protocol. Reverse transcription was performed using a miR‐125a‐5p‐specific primer and ABI's TaqMan MicroRNA Reverse Transcription kit (Applied Biosystems, Thermo Fisher Scientific). miR‑125a‐5p expression level was detected using a Taqman MicroRNA assay (Applied Biosystems, Thermo Fisher Scientific) with the Applied Biosystems 7900HT Sequence Detection system. U6 was used as the internal control. The RT‐qPCR thermocycling conditions were as follows: 94°C for 30 s (initial denaturation), 94°C for 5 s (denaturation) and 55°C for 30 s (annealing), for 40 cycles. The following primers were used: miR‐125a‐5p forward, 5′‐GGTAAGTCACGCGGT‐3′ and reverse, 5′‐CAGTGCGTCTCGTGGAGT‐3′; U6 forward, 5′‐CTGGTTAGTACTTGGACGGGAGAC‐3′ and reverse, 5′‐GTG CAGGGTCCGAGGT‐3′. Subsequently, the 2^−ΔΔ^Cq method was used to quantify the expression level of the miRNA relative to U6.

The article "Epigenetic silenced miR‐125a‐5p could be self‐activated through targeting Suv39H1 in gastric cancer" was retracted in 2021. Reasons: errors in the data; errors in the images; unreliable results or conclusions; concerns about a third party's involvement.

### 2.3 DNA extraction and methylation analysis

Genomic DNA was isolated from tissues or cultured cells using the Universal Genomic DNA Extraction Kit Ver. 3.0 (Takara) in accordance with the manufacturer's instructions. The quality and integrity of DNA were checked by electrophoresis on 1% agarose gel, quantified spectrophotometrically. Bisulphite modification of DNA was produced by using the EpiTect Bisulfite Kit (Qiagen) according to the manufacturer's recommendations. In brief, the DNA (1 μg) was denatured using NaOH and subsequently modified by sodium bisulphite. Then, the mixture was desulfonated, and DNA was purified on silica‐membrane columns. The bisulphite‐treated miR‐125a‐5p promoter regions containing CpG sites was amplified and subcloned into a pGEM T‐Easy vector (Promega) after gel purification. The resulting products were next transformed into JM109 competent cells. Methylation states of each CpG site were analysed by randomly sequencing 10 clones. The methylation level for each sample was calculated as the percentage of methylated CpG dinucleotides from the total number of CpG dinucleotides.

### 2.4 Cell culture and transfection

Primary gastric cancer cell line GC‐114 and GC‐026 were isolated from gastric cancer tissues. The cell line HEK293T and gastric cancer cell line NCI‐N87 were purchased from China Center for type culture collection in Wuhan. All cells were cultured with RPMI‐1640 medium (Gibco) containing 10% foetal bovine serum (FBS) (Gibco). MicroRNA was transfected at 30 nmol/L (final concentration) using Lipofectamine^™^ RNAiMAX (Thermo Fisher Scientific) according to the manufacturer's instructions.

### 2.5 Luciferase reporter assay

The 3′‑UTR of human Suv39H1 containing the potential miR‐125a‐5p binding sites was amplified by high fidelity PCR. Then, the amplified sequence was cloned into the XbaI site of the pGL3 control vector (Promega). The mutated putative miR‐125a‐5p binding site in the 3′‐UTR of Suv39H1 was generated using the QuickChange Site‐directed Mutagenesis kit (Stratagene) according to the manufacturer's protocol. The day before transfection, HEK293T cells were seeded in 24‐well plates (5 × 10^4^ cells/well), then we transfected 500 ng Suv39H1 3′‐UTR‐pGL3 and 30 nmol/L (final concentration) miR‐125a‐5p mimics or control miRNA mimics (Ambion) into the cells with Lipofectamine 2000. Forty‐eight hours after transfection, luciferase activity was determined using dual‐luciferase reporter assay system (Promega) according to the manufacturer's protocol.

The article "Epigenetic silenced miR‐125a‐5p could be self‐activated through targeting Suv39H1 in gastric cancer" was retracted in 2021. Reasons: errors in the data; errors in the images; unreliable results or conclusions; concerns about a third party's involvement.

### 2.6 Western blotting

Total protein from tumour tissues or cultured cells was lysed in RIPA buffer with protease inhibitor (Beyotime, Shanghai, China). The protein was quantified using a BCA assay kit (Beyotime, Shanghai, China). A total of 20 μg of total protein were separated by 10% SDS‐PAGE, transferred onto polyvinylidene fluoride membranes and then reacted with primary antibodies against Suv39H1, H3K9me3 and β‐actin (Abcam). After being extensively washed with PBS containing 0.1% Triton X‐100, the membranes were incubated with alkaline phosphatase‐conjugated goat anti‐rabbit antibody for 30 minutes at room temperature. The bands were visualized using 1‐step TM NBT/BCIP reagents (Thermo Fisher Scientific, Rockford, IL) and detected by an Alpha Imager (Alpha Innotech, San Leandro, CA).

### 2.7 Cell viability assay

Cell viability was evaluated using CCK‐8 (Beyotime, Shanghai, China) according to manufacturer's instructions. Briefly, cells were seeded into 96‐well plates at 5 × 10^3^ cells per well and cultured for indicated time points. Ten microlitres of CCK‐8 solution was added into the culture medium in each well. After 1‐hour incubation, OD values were read using a microplate reader (Bio‐Tek Company, Winooski, VT, USA) at the 450‐nm wavelength. Each time point was repeated in three wells, and the experiment was independently performed for three times.

### 2.8 Cell apoptosis assay

Cell apoptosis was evaluated by flow cytometry using an Annexin V‐FITC Apoptosis Detection Kit (KeyGen Biotech Co. Roche, Nanjing, China). Briefly, cells were seeded into 24‐well plates at 1 × 10^5^ cells per well and cultured for 48 hours. Then, the cells were detached by trypsinization, washed twice in PBS (400 g, 5 minutes; Allegra X‐12R centrifuge; Beckman Coulter, USA) and resuspended in 500 μL binding buffer. A volume of 5 μL Annexin V‐FITC and 5 μL propidium iodide was added and mixed gently, and the cells were stained in the dark for 10 minutes at room temperature. The cells were analysed immediately by flow cytometry (BD FACSCalibur, BD Bioscience, San Diego, CA, USA) and analysed using Flowjo software (FlowJo, Ashland, OR, USA). The experiment was repeated three times.

### 2.9 Cell migration assay

The migration of cells was detected by wound‐healing assay. Cells were cultured in 6‐well plates. When the cells grew to 80%‐90% confluence, a wound in a line across the well was made by a plastic pipette tip. The area of cell‐free wound was recorded 24 hours later using an inverted microscope and analysed by the NIH Image 1.55 software. Wound healing = 100× (1‐the remaining cell‐free area/the area of the initial wound). All tests were performed in triplicate.

The article "Epigenetic silenced miR‐125a‐5p could be self‐activated through targeting Suv39H1 in gastric cancer" was retracted in 2021. Reasons: errors in the data; errors in the images; unreliable results or conclusions; concerns about a third party's involvement.

### 2.10 Transwell invasion assay

Invasive ability of cells was determined within a transwell system. 6.0 × 10^4^ cells were seeded onto the upper surface of the transwell membrane and cultured at 37°C in 5% CO_2_ for 24, 48 and 72 hours.The number of cells that migrated to the lower surface of the membrane was counted under a microscope (200×).

### 2.11 Lentivirus preparation

The miR‐125a‐5p was cloned into lentiviral pLKO.1‐puro vector and the empty vector as negative control. Lentiviruses were prepared using HEK293T cells according to the manufacturer's instructions. GC‐026 cells were incubated with lentivirus and 4 mg/mL polybrene (AmericanBio) for 24 hour.

### 2.12 Animal study

Six‐ to week‐old NOD/SCID mice (Charles River Laboratories, Beijing, China) were housed in specific pathogen‐free conditions. The study was approved by the Research Ethics Committee of Zhangzhou Affiliated Hospital of Fujian Medical University. Mice were housed in the pathogen‐free region and monitored daily during the experiments, and the mice would be sacrificed when the weight loss is more than 20%. For evaluation of the tumour growth in vivo, 5 × 10^6^ GC‐026 cells were suspended in 200 μL PBS and injected subcutaneously into the dorsal scapula region of the mice. Four weeks later, the tumour size was measured with fine digital callipers and calculated by the following formula: tumour volume = 0.5 × width^2^ × length.

### 2.13 Statistical analysis

Data were expressed as mean ± SE and analysed by a SPSS software package (SPSS Standard version 13.0, SPSS Inc, USA). Differences between variables were assessed by the chi‐square test. Survival analysis of patients with colorectal cancer was calculated by Kaplan–Meier analysis. A log rank test was used to compare different survival curves. A Cox proportional hazards model was used to calculate univariate and multivariate hazard ratios for the variables. Unpaired Student's *t* test and one‐way ANOVA were used as appropriate to assess the statistical significant of difference. *P* values under .05 were considered statistically significant.

## 3 RESULTS

### 3.1 Decreased miR‐125a‐5p level in gastric cancer biopsies

A total of 286 cases with gastric cancer were followed. All these patients had received no pre‐operation chemotherapy. They were given the same radical operation and underwent the same adjuvant chemotherapy after the surgery. The miR‐125a‐5p level was firstly analysed and the data showed that the miR‐125a‐5p level reduced significantly in gastric cancer tissues comparing with its paired adjacent non‐cancerous tissues (Figure 1A). The reduced miR‐125a‐5p level was associated with tumour size (*P *=* *.001), lymph node (*P *=* *.009) and liver metastasis (*P *=* *.012, Table 1).

The article "Epigenetic silenced miR‐125a‐5p could be self‐activated through targeting Suv39H1 in gastric cancer" was retracted in 2021. Reasons: errors in the data; errors in the images; unreliable results or conclusions; concerns about a third party's involvement.

**Figure 1:** Reduced miR‐125a‐5p is correlated with the poor prognosis of gastric cancer. A, miR‐125a‐5p levels in cancer tissues and adjacent normal tissues were determined by qPCR (n = 286). Result is depicted as box plots; middle line indicates median; bottom of box, 25th percentile; and top of box, 75th percentile. *P <* *.05. B, Kaplan–Meier survival curve of patients with high or low level of miR‐125a‐5p. C, miR‐125a‐5p methylation levels in cancer tissues and adjacent normal tissues were determined (n = 286). Result is depicted as box plots; middle line indicates median; bottom of box, 25th percentile; and top of box, 75th percentile. *P <* *.05. D, Correlation between the mRNA level and the methylation level of miR‐125a‐5p. *Inset* corresponds to Pearson's *R* correlation and corresponding *P* value

Disease‐free survival (DFS) and overall survival (OS) were conducted to assess the predictive role of miR‐125a‐5p level for metastasis. Both DFS and OS were significantly higher in the high miR‐125a‐5p level group than the low miR‐125a‐5p level group (Figure 1B). The low miR‐125a‐5p level group subsequently developed more metastasis than the high miR‐125a‐5p level group (*P *<* *.05, Table 1). Univariate and multivariate analysis showed that patients with reduced miR‐125a‐5p level had a significantly reduced OS and DFS (Tables 2 and 3).

**Table 2:** Univariate Cox proportional hazards model for disease‐free survival (DFS) and overall survival (OS)

	DFS			OS		
	HR	95% CI	*P* value	HR	95% CI	*P* value
Age, y						
<65	—			—		
≥65	1.009	0.659‐1.841	.714	0.934	0.530‐1.644	.812
Differentiation						
Well	—			—		
Moderate	0.816	0.309‐2.155	.681	0.789	0.267‐2.334	.669
Low	1.251	0.718‐2.176	.431	1.145	0.614‐2.135	.671
Tumour size, cm						
<50 mm (small)	—			—		
≥51 mm (large)	5.887	3.025‐11.456	<.001^a^	4.157	2.009‐8.602	<.001^a^
Lymph node metastasis						
Yes	4.315	0.750‐12.306	.041^a^	4.458	0.764‐12.780	.023^a^
No	—			—		
Liver metastasis						
Yes	4.901	2.469‐9.721	<.001^a^	4.638	2.152‐9.997	<.001^a^
No	—			—		
miR‐125a‐5p						
High	—			—		
Low	6.118	3.004‐12.462	<.001^a^	6.348	2.875‐14.014	<.001^a^

a *P *<* *.05 indicates a significant association among the variables.

**Table 3:** Multivariate Cox proportional hazards model for DFS and OS

	DFS			OS		
	HR	95% CI	*P* value	HR	95% CI	*P* value
Lymph node metastasis	2.796	1.919‐4.161	<.001^a^	2.659	1.711‐4.223	<.001^a^
Liver metastasis	1.701	1.129‐2.541	.008^a^	3.981	1.854‐9.173	<.001^a^
miR‐125a‐5p level	4.402	1.299‐14.551	.011^a^	8.001	2.403‐26.815	<.001^a^

a *P *<* *.05 indicates a significant association among the variables.

The article "Epigenetic silenced miR‐125a‐5p could be self‐activated through targeting Suv39H1 in gastric cancer" was retracted in 2021. Reasons: errors in the data; errors in the images; unreliable results or conclusions; concerns about a third party's involvement.

It has been demonstrated that the epigenetic modulators could modulate the miR‐125‐5p expression,^13^, ^25^, ^26^ and its promoter is hypermethylated in glioma cells.^27^ We analysed the miR‐125a‐5p methylation status in gastric cancer tissues and adjacent non‐tumour tissues. We designed and validated bisulphate sequencing PCR for the promoter region of miR‐125a‐5p including 20 CpGs. Data showed that the miR‐125a‐5p was hypermethylated in gastric cancer tissues comparing with the adjacent non‐cancer tissues (Figure 1C). To further determine whether DNA methylation contributes to the silencing of miR‐125a‐5p in gastric cancer, the correlation between the miR‐125a‐5p and its methylation level was analysed. And the methylation status was negatively correlated with its expression level (Figure 1D).

Taken together, the data showed that the epigenetic silenced miR‐125a‐5p might contribute to gastric cancer development and the poor outcomes.

### 3.2 Suv39H1 is directly regulated by miR‐125a‐5p

To uncover the potential mechanism of the epigenetic silencing of miR‐125a‐5p in gastric cancer cells, the potential targets of miR‐125a‐5p were screened using prediction tools including miRanda, TargetScan and Pictar algorithms. Among the hundreds of targets that were predicted, the histone methyltransferase Suv39H1 was further studied. To obtain the direct evidence that Suv39H1 is a potential target of miR‐125a‐5p, we examined whether the predicted binding sites of miR‐125a‐5p in the 3′‐UTR of Suv39H1 mRNA were responsible for its regulation (Figure 2A). The 3′‐UTR of Suv39H1 was cloned into the downstream of a luciferase reporter, and this vector was co‐transfected with an miR‐125a‐5p mimic or its negative control into HEK293T cells. The luciferase activity of cells transfected with miR‐125a‐5p mimic was significantly reduced compared with the negative control (*P *<* *.05; Figure 2B). Furthermore, deletion of the putative binding site clearly abrogated the repression of luciferase activity caused by miR‐125a‐5p overexpression (Figure 2B).

**Figure 2:** Suv39H1 is the miR‐125a‐5p target gene. A, The potential binding site of miR‐125a‐5p in the 3′UTR of Suv39H1. B, Luciferase assay performed by overexpressing miR‐125a‐5p and the wild type of Suv39H1 3′UTR (WT‐3′UTR) or the 3′UTR without potential miR‐125a‐5p binding site (Mut‐3′UTR). n = 3. *P <* *.05. C, Suv39H1 levels in cancer tissues and adjacent normal tissues were determined by qPCR (n = 286). Result is depicted as box plots; middle line indicates median; bottom of box, 25th percentile; and top of box, 75th percentile. *P <* *.05. D, Overexpressing miR‐125a‐5p could suppress the Suv39H1 expression in two primary gastric cancer cell line (GC‐114 and GC‐026), determined by qPCR. n = 3. *P <* *.05. E, Overexpressing miR‐125a‐5p could suppress the Suv39H1 expression in two primary gastric cancer cell line (GC‐114 and GC‐026), determined Western blot. NC: empty vector. F, Cell morphology of the primary gastric cancer cell line GC‐114 and GC‐026

If the Suv39H1 is regulated by miR‐125a‐5p in gastric cancer, the Suv39H1 expression level in gastric cancer tissue should be up‐regulated as the down‐regulation of miR‐125a‐5p. As expected, the mRNA level of Suv39H1 was up‐regulated in gastric cancer tissue comparing with the adjacent non‐tumour tissues (Figure 2C). This was further validated in two primary isolated gastric cancer cell lines: GC‐114 and GC‐026. After overexpressing miR‐125a‐5p, the mRNA and protein levels of Suv39H1 were suppressed significantly (Figure 2D,E). This was further validated in the well established gastric cancer cell line NCI‐N87 (Figure S1).

The article "Epigenetic silenced miR‐125a‐5p could be self‐activated through targeting Suv39H1 in gastric cancer" was retracted in 2021. Reasons: errors in the data; errors in the images; unreliable results or conclusions; concerns about a third party's involvement.

These data suggested that miR‐125a‐5p might inhibit the Suv39H1 expression through 3′‐UTR in gastric cancer tissues, and affect the epigenetic status of the cancer cells.

### 3.3 Demethylation and activation of endogenous miR‐125a‐5p through exogenous overexpressing miR‐125a‐5p

Because Suv39H1 is a histone‐lysine N‐methyltransferase that specifically trimethylates Lys‐9 of histone H3 (H3K9me3), we first determined whether overexpressing miR‐125a‐5p would affect the H3K9 trimethylation (H3K9me3) status through targeting Suv39H1. As expected, the whole genome H3K9me3 level was decreased after overexpressing miR‐125a‐5p (Figure 3A). The H3K9me3 is also tightly related to the DNA methylation. Thus, we then measured the miR‐125a‐5p methylation level after miR‐125a‐5p overexpression. Interestingly, the methylation level was decreased by overexpressing miR‐125a‐5p (Figure 3B). Furthermore, the endogenous miR‐125a‐5p precursor was also up‐regulated (Figure 3C). This up‐regulation and demethylation of miR‐125a‐5p were abolished when overexpressing miR‐125a‐5p and Suv39H1 together (Figure 3D‐F), indicating that miR‐125a‐5p could modulate its own methylation and expression through Suv39H1. This was further validated in the well‐established gastric cancer cell line NCI‐N87 (Figure S2).

**Figure 3:** Demethylation and activation of endogenous miR‐125a‐5p through exogenous overexpressing miR‐125a‐5p. A, Overexpressing miR‐125a‐5p could suppress the H3K9me3 level in two primary gastric cancer cell line (GC‐114 and GC‐026), determined by Western blot. B, Overexpressing miR‐125a‐5p could suppress the miR‐125a‐5p methylation levels in two primary gastric cancer cell line (GC‐114 and GC‐026). n = 3. *P <* *.05. C, Overexpressing miR‐125a‐5p could up‐regulate the endogenous miR‐125a‐5p precursor expression in two primary gastric cancer cell line (GC‐114 and GC‐026), determined by qPCR. n = 3. *P <* *.05. D, Successful overexpression of Suv39H1 in two primary gastric cancer cell line (GC‐114 and GC‐026), determined by Western blot. E, Up‐regulation of endogenous miR‐125a‐5p precursor by exogenous miR‐125a‐5p overexpression could be abolished by Suv39H1 overexpression in two primary gastric cancer cell line (GC‐114 and GC‐026), determined by qPCR. n = 3. *P <* *.05. F, The demethylation of miR‐125a‐5p by exogenous miR‐125a‐5p overexpression could be abolished by Suv39H1 overexpression in two primary gastric cancer cell line (GC‐114 and GC‐026). n = 3. *P <* *.05. NC: empty vector

The article "Epigenetic silenced miR‐125a‐5p could be self‐activated through targeting Suv39H1 in gastric cancer" was retracted in 2021. Reasons: errors in the data; errors in the images; unreliable results or conclusions; concerns about a third party's involvement.

### 3.4 Overexpression of miR‐125a‐5p inhibits gastric cancer cell activities

It has been demonstrated that miR‐125a‐5p functions as tumour suppressor and our data also showed that its expression decreased in the gastric cancer specimens. Thus, we further evaluated the anti‐tumour effects of miR‐125a‐5p in vitro. Two gastric cancer cell lines isolated from gastric cancer specimens were used. And our data showed that overexpressing miR‐125a‐5p could inhibit the gastric cancer cell migration (Figure 4A), invasion (Figure 4B) and proliferation (Figure 4C). In addition, the miR‐125a‐5p could accelerate the gastric cancer cell apoptosis (Figure 4D). This was further validated in the well‐established gastric cancer cell line NCI‐N87 (Figure S3).

**Figure 4:** Increasing miR‐125a‐5p levels suppressed gastric cancer cell activities. A, Wound‐healing assay with overexpressing miR‐125a‐5p or empty vector (NC) in two primary gastric cancer cell line (GC‐114 and GC‐026). n = 3. *P <* *.05. B, Cell invasion assay with overexpressing miR‐125a‐5p or empty vector (NC) in two primary gastric cancer cell line (GC‐114 and GC‐026). n = 3. *P <* *.05. C, The survival rate analysis with overexpressing miR‐125a‐5p or empty vector (NC) in two primary gastric cancer cell line (GC‐114 and GC‐026). n = 3. *P <* *.05. D, The cell apoptosis analysis with overexpressing miR‐125a‐5p or empty vector (NC) in two primary gastric cancer cell line (GC‐114 and GC‐026). n = 3. *P <* *.05

### 3.5 Overexpressing miR‐125a‐5p suppresses gastric cancer development in vivo

To further confirm the important role of miR‐125a‐5p level on gastric cancer development, human gastric cancer cell line GC‐026 was firstly infected with lentivirus expressing miR‐125a‐5p. Then, the cells were transplanted subcutaneously into the dorsal scapula region of the NOD/SCID mice. Data showed that overexpressing miR‐125a‐5p inhibited gastric cancer development in vivo (Figure 5A). Furthermore, exogenous miR‐125a‐5p overexpression could decrease the endogenous miR‐125a‐5p methylation level (Figure 5B) and also promotes its precursor expression (Figure 5C). The Suv39H1 level was also decreased after miR‐125a‐5p overexpression (Figure 5D). These data showed that overexpressing miR‐125a‐5p inhibited gastric cancer development in vivo through suppressing Suv39H1 expression, resulting in endogenous miR‐125a‐5p demethylation and up‐regulation.

The article "Epigenetic silenced miR‐125a‐5p could be self‐activated through targeting Suv39H1 in gastric cancer" was retracted in 2021. Reasons: errors in the data; errors in the images; unreliable results or conclusions; concerns about a third party's involvement.

**Figure 5:** Overexpressing miR‐125a‐5p suppressed gastric cancer development in vivo. A, Overexpressing miR‐125a‐5p decreased the tumour size in vivo. n = 12. *P <* *.05. B, Overexpressing miR‐125a‐5p decreased the methylation level of miR‐125a‐5p in vivo. n = 12. *P <* *.05. C, Overexpressing miR‐125a‐5p increased the expression of endogenous miR‐125a‐5p precursor in vivo. n = 12. *P <* *.05. D, Overexpressing miR‐125a‐5p suppressed the expression of Suv39H1 in vivo. n = 12. *P <* *.05. NC: empty vector

## 4 DISCUSSION

MicroRNAs (miRNAs) are a class of single‐stranded non‐coding RNAs that regulate target gene expression, predominantly by base pairing to the 3′‐untranslated (3′‐UTR) region of their target mRNAs.^4^, ^5^, ^6^ Recent studies have established the presence of miRNA expression signatures in gastric cancer, but our understanding of the function of aberrant miRNAs in gastric cancer progression remains in its infancy.^3^, ^7^, ^8^

miR‐125a‐5p has been previously reported to be down‐regulated in various human cancer types, including gastric cancer.^9^, ^20^, ^21^, ^22^ Furthermore, miR‐125a‐5p has been validated to prevent the cancer cell progression.^10^, ^11^, ^12^, ^13^, ^14^, ^15^, ^16^, ^17^, ^18^, ^19^, ^23^, ^24^ However, the underlying mechanism of the low expression of miR‐125a‐5p in gastric cancer remains unknown.

In the present study, it was further confirmed that the miR‐125a‐5p expression was reduced in most gastric cancer tissues comparing with the adjacent non‐tumour tissues. And the down‐regulation was tightly correlated with the low overall survival and disease‐free survival. DNA methylation analysis showed that the miR‐125a‐5p promoter was highly methylated and negatively associated its expression. Aberrant promoter methylation is considered a hallmark of cancer involved in silencing of tumour suppressor genes and activation of oncogenes. Aberrant DNA methylation includes hyper/hypomethylation. For tumour suppressor genes, such as miR‐125a‐5p, the molecules are commonly hypermethylated in tumour tissues compared with non‐tumour tissues. In addition to our study here, the miR‐125a‐5p has been demonstrated to be hypermethylated in glioma cells.^27^

The article "Epigenetic silenced miR‐125a‐5p could be self‐activated through targeting Suv39H1 in gastric cancer" was retracted in 2021. Reasons: errors in the data; errors in the images; unreliable results or conclusions; concerns about a third party's involvement.

Target gene screening and validation showed that the histone methyltransferase Suv39H1 was the miR‐125a‐5p target gene, which was also involved into the epigenetic silencing of the miR‐125a‐5p. It has been demonstrated that Suv39H1 is overexpressed in gastric cancers and knocking‐down Suv39H1 could suppress gastric cancer development, which is in accordance with our results here.^28^ In addition to the interactions between epigenetic modulation by Suv39H1 and miR‐125a‐5p uncovered in the current study, it has also been demonstrated HDACs and Sirtuins are also involved into this process.^13^, ^25^, ^26^ Overexpessing miR‐125a‐5p could self‐activate the silenced miR‐125a‐5p in gastric cancer cells, resulting in cancer suppression in vitro and in vivo. The data here showed that the miR‐125a‐5p might be not only the potential prognostic value as a tumour biomarker but also potential therapeutic targets in gastric cancer.

The identification of the expression levels and tumour suppressive function of miR‐125a‐5p in gastric cancer provides a new window of therapeutic opportunity. The development of modified miRNAs with longer half‐time and higher efficiency has produced favourable anticancer outcomes in experimental models, including the locked nucleic acid modified oligonucleotides and the antisense oligonucleotides.^4^, ^5^, ^6^ Therefore, enforced expression of miR‐125a‐5p utilizing approaches such as transfection of miR‐125a‐5p‐carrying viruses or synthetic miR‐125a‐5p oligos will be required for future study in gastric carcinoma pathology.

## CONFLICT OF INTEREST

The authors declare that they have sno competing interests.
